# Capecitabine and bevacizumab for non-resectable metastatic colorectal cancer patients: final results from phase II AIO KRK 0105 trial

**DOI:** 10.1186/1471-2407-13-454

**Published:** 2013-10-04

**Authors:** Alexander Stein, Albrecht Kretzschmar, Dirk Behringer, Thomas Wolff, Joachim Zimber, Susanna Hegewisch-Becker, Erika Kettner, Karl-Heinz Pflüger, Andreas Kirsch, Dirk Arnold

**Affiliations:** 1 University Medical Center, Hamburg-Eppendorf, Hamburg, Germany; 2 Krankenhaus St Georg, Leipzig, Germany; 3 Augusta-Kranken-Anstalt, Bochum, Germany; 4 Praxis Lerchenfeld, Hamburg, Germany; 5 Praxis, Nürnberg, Germany; 6 Onkologische Schwerpunktpraxis Eppendorf, Hamburg, Germany; 7 University of Magdeburg, Universitätsplatz 2, 39106 Magdeburg, Germany; 8 Evangelisches Diakonie-Krankenhaus gGmbH, Bremen, Germany; 9 Praxis Oskar Helene Heim, Berlin, Germany; 10 Tumor Biology Center Freiburg, Breisacher Str. 117, 79106 Freiburg, Germany

**Keywords:** Non-resectable, Metastatic, Colorectal cancer, Capecitabine, Bevacizumab

## Abstract

**Background:**

Current guidelines recommend treatment with capecitabine and bevacizumab for patients (pts) with non-resectable metastatic colorectal cancer (mCRC), although clinical data in this particular patient group are lacking.

**Methods:**

Previously untreated patients with non-resectable mCRC were to receive capecitabine (1,250 mg/sqm bid d1-14 oral) and bevacizumab (7.5 mg/kg i.v.) every 3 weeks. Progression-free survival (PFS) was the primary endpoint. Secondary endpoints include overall survival (OS), objective response rate (ORR) and toxicity.

**Results:**

82 pts were included: 40 female, median age 70 (range 50–86). ECOG PS 0/1/2 was 38/52/10%, respectively. Synchronous metastases were present in 58 pts. 16 pts had primary tumor in situ. Median treatment duration was 4.1 months (6 cycles). Toxicity was generally mild. ORR was 38%, with 5 complete and 23 partial responses. Median PFS was 7.0 months [95% CI (5.0-9.1)] and OS 17.9 months [95% CI (14.6-21.6)]. Second- and third-line systemic therapy was given to 57% and 33% of pts, respectively.

**Conclusions:**

Besides the favourable tolerability, PFS and OS were shorter than reported by other trials. Careful patient selection for upfront capecitabine and bevacizumab is essential.

## Background

Colorectal cancer (CRC) is the most frequently diagnosed cancer in Europe and one of the leading causes of cancer death worldwide [1,2]. Several first-line treatment options for metastatic CRC (mCRC) are currently available, incorporating fluoropyrimidines, irinotecan, oxaliplatin, bevacizumab and epidermal growth factor receptor (EGFR) antibodies (i.e. cetuximab and panitumumab) for (K)RAS wildtype patients [3-8].

Current guidelines recommend first line single agent fluoropyrimidine with or without bevacizumab for patients without an option for resection, either due to location or comorbidity, and asymptomatic/low volume disease (so called group 3 patients) [9]. The combination of 5-fluorouracil and bevacizumab was established by two randomized phase II trials, demonstrating prolonged progression free (PFS) and overall survival (OS) and higher objective response rates (ORR) for the addition of bevacizumab to a bolus regimen of 5-fluorouracil and leucovorin (5FU/LV) [10,11]. These trials included either unselected patients or patients considered to be not optimal candidates for first line irinotecan. At the time of initiation of the current study no prospectively collected data of the combination of the oral fluoropyrimidine capecitabine and bevacizumab were available.

Later the Australasian Gastrointestinal Trials Group (AGITG) MAX trial evaluated capecitabine +/− bevacizumab, with a third arm adding mitomycin, in patients suitable for capecitabine single agent. The combination of capecitabine and bevacizumab showed significantly prolonged PFS (8.5 vs. 5.7 months, hazards ratio (HR) 0.63; p = 0.03) and a beneficial trend for OS and ORR [12].

Moreover, several single arm phase II trials and a randomized phase III trial were applying capecitabine and bevacizumab in elderly patients (≥70 years of age) [13-16]. In this particular patient group capecitabine and bevacizumab was feasible and efficacious with a response rate of about 20% and a median PFS of 9.1-11.5 months. Despite the recommendation, data on the use of capecitabine and bevacizumab in definitely non-resectable patients independent of appropriateness for intensive first line treatment are scarce.

## Methods

### Patient selection

Patients were required to have a histological confirmed diagnosis of mCRC not amenable for upfront or secondary resection (defined as no option for curative treatment either initially or after reduction in size of metastases after chemotherapy), Eastern Cooperative Oncology Group performance status of 0–2, measurable disease according to Response Evaluation Criteria in Solid Tumors (RECIST) version 1.0 and adequate hematological, renal, and hepatic function defined by the following criteria: neutrophil count ≥1500/mm3, platelet count ≥ 100 000/mm3, creatinine-clearance ≥ 30 ml/min, total serum bilirubin ≤ 2 times the upper limit of the institutional normal range (ULN), and transaminases ≤ 2,5 times ULN. Exclusion criteria included prior chemotherapy for metastatic disease (adjuvant chemotherapy completed at least 6 months before trial inclusion was allowed); other active malignancy within the preceding year except for adequately treated basal cell cancer, or in situ cervical cancer; clinical evidence of central nervous system - metastases; major operation or injury within 28 days; and clinically significant cardiovascular disease.

All patients provided written informed consent before study entry according to institutional regulations. The trial was approved by the institutional review board and the competent authority (Paul Ehrlich Institut) and registered (EudraCT number: 2005-001919-21).

### Treatment administration

All patients received capecitabine and bevacizumab in a 3-weekly cycle. Capecitabine was administered with 1250 mg/m^2^ body surface area orally twice-daily days 1–14. The daily dose of capecitabine was calculated to the next 500 mg dose level. If the calculated dose was < 400 mg above the last 500 mg dose level, it was rounded down. If it was ≥ 400 mg above it, it was rounded up to the next 500 mg dose level. Bevacizumab was administered with 7.5 mg/kg body weight as an intravenous infusion on day 1.

### Dose adjustments

New treatment cycle was scheduled if neutrophil count was ≥ 1500/mm3, platelet count was ≥ 100 000/mm3, and all relevant non-hematological toxic effects were grade 1 or lower (NCI CTC AE v 3.0). Dose reductions were based on the toxicity in the preceding cycle. Capecitabine doses were reduced by 25% for any grade 3 or 4 hematological toxicity, except anemia. Treatment was held for grade 3 non-hematological adverse events (excluding alopecia, nausea or vomiting), until resolution to grade 1 or lower, and resumed at a 25% reduction and discontinued for grade 4 non-hematological adverse. In case of a drug specific adverse event, e.g. hand-foot syndrome for capecitabine the suspected drug was reduced. Capecitabine was reduced by 25% for mild renal impairment with creatinine clearance from 30 to 50 ml/min. Patients requiring a treatment delay of more than 2 weeks due to toxicity or more than two dose reductions were removed from the study. In addition, patients were removed from study for disease progression, unacceptable toxicity, or withdrawal of consent.

### Study evaluations

Pretreatment evaluation included a complete medical history, physical examination, routine hematology, biochemistry and urine analyses, and computed tomography (CT) scans of the abdomen and pelvis and thoracic CT scan in case of pulmonary metastases. Hematological (including platelet and differential) analyses, serum chemistry, and urine dipstick were obtained at day 1 in each cycle. Subjective symptoms, physical examination results, vital signs (including blood pressure), performance status, and all adverse reactions were recorded before each treatment cycle according to NCI CTC AE v 3.0. CT scans were performed every 9 weeks (three cycles) to assess disease status. Response rate was evaluated according to RECIST 1.0 [17].

### Statistical considerations

The primary end point of this phase II trial was progression free survival rate at 9 months (PFSR@9). A single-stage study design was planned. The primary goal was to demonstrate a PFSR@9 of at least 50%, similarly to the efficacy reported with 5FU/LV and bevacizumab. Treatment with capecitabine and bevacizumab would however be seen as insufficiently effective if PFSR@9 would be not more than 35% (which corresponds to a progression-free survival of 6 months). With 85% power and one-sided type I error of 0.05 the required sample size was 76 patients. With a drop out rate of 5%, 82 patients were to be included. Baseline patient characteristics, response, and toxic effects were described using summary statistics. The Kaplan-Meier-method was used to analyze the primary endpoint and censored event times. 95%-confidence intervals (CI) were given for all calculated estimates.

## Results

### Patients’ characteristics

Between December 2006 and September 2008, a total of 82 patients were enrolled at 20 German study sites. 4 patients did not receive any study treatment and were withdrawn prior to administration of study drug (due to infection, progression or protocol deviation) and are thus not included in the safety population. Baseline characteristics are summarized in Table 1. 40 female and 42 male patients with median age of 70 years (range 49–86 years) and ECOG PS score of 0/1/2 in 38/52/10% respectively were analyzed. Site of primary tumor was colon in 56 and rectum in 26 patients. Synchronous metastatic disease was present in 58 (72%) patients. Prior resection of primary tumor was performed in 66 (80%) patients.

**Table 1:** Patients’ characteristics

**Characteristic**	**n**	**%**	**Years**
Age: median (range)			70 (49–86)
Sex			
Female	40	49	
Male	42	51	
ECOG			
0	31	38	
1	43	52	
2	8	10	
Comorbidity (clinically relevant)			(1 missing)
yes	66	81	
**Primary tumor**			
Colon	56	68	
Rectum	26	32	
Resected primary tumor	66	80	
Prior radiotherapy for rectal primary	12	15	
Adjuvant chemotherapy	19	23	
**Metastases**			(1 missing)
synchronous metastases	58	72	
metastatic sites			
1	34	42	
>1	47	58	
liver metastases	65	80	
**Prognosis score acc. to Kohne et al.**			(8 missing)
low risk	64	86	
high risk	10	14	

*Abbreviations*: ECOG Eastern Cooperative Oncology Group performance status, n number.

### Treatment received

A total of 607 cycles was administered, with a median number of 6 (range 1–24) cycles per patient. Median treatment duration was 4.1 months (range 0.1-17.5) (for bevacizumab 3.7 months). Dose reductions were adopted in 15% of the documented cycles and were mainly related to capecitabine. Bevacizumab dose was only reduced in less than 1% of the cycles. Overall 44 patients (56%) had to be dose reduced. Treatment was delayed in 18% of cycles. Reason for discontinuation of study treatment were progressive disease in 41 (53%), toxicity in 8 (10%), withdrawal of consent in 5 (6%), death (other than tumor) 5, protocol violation 2, resection/radiotherapy/local ablation in 3 patients and unknown in 18 patients. Second- and third-line treatments were administered to 47 and 27 patients (57% and 33%), respectively. Oxaliplatin and irinotecan were applied in 29 and 35 patients (35% and 43%), respectively, with only 17 patients (21%) receiving both drugs consecutively. Salvage treatment with EGFR antibodies was performed in 17 patients (21%), mostly combined with irinotecan (10 patients).

### Efficacy

The efficacy results were determined in the group of patients receiving at least one treatment (n = 78). Results are summarized in Table 2. Progression free survival rate at 9 months was 0.35 [95% CI (0.24-0.46)]. Objective response rate (ORR) was 38% with 5 complete (7%) and 23 partial responses (31%). Stable disease as best response was achieved in 31 patients (43%), resulting in a disease stabilisation rate of 81%. After a median follow up of 12.7 months, median PFS was 7.0 months [95% CI (5.0-9.1)] (Figure 1) and median OS was 17.9 months [95% CI (14.6-21.6)] (Figure 2). The 1-year overall survival rate was 67% [95% CI (56–79)]. The median duration of response, defined as PFS of the subgroup of 28 patients achieving objective response, was 8.9 months [95% CI (8.0-14.6)]. The median time to documentation of objective response in this subgroup was 3.4 months.

**Table 2:** Efficacy according to RECIST 1.0

**Efficacy in patients receiving treatment (n = 78)**			
	**n**	**%**	
Response rate (evaluable n = 73)			(5 missing)
Complete response	5	7	
Partial response	23	31	
Stable disease	31	43	
Progressive disease or death	14	19	
		**95% CI**	
PFS rate at 9 months	0.35	0.24-0.46	
PFS	7.0 months	5.0-9.1	
OS	17.9 months	14.6-21.6	

*Abbreviations*: n number, PFS Progression free survival, OS Overall survival, CI Confidence interval.

**Figure 1:** Kaplan–Meier survival curve demonstrating progression-free survival.

**Figure 2:** Kaplan–Meier survival curve demonstrating overall survival.

### Toxicity

Treatment was generally well tolerated in an outpatient setting. Adverse events are summarized in Table 3. The most frequently observed adverse event were hand-foot skin reaction (57% of patients) and infection (37%). 16 patients (21%) experienced grade 3 hand-foot skin reaction. Hypertension occurred in 17 patients (22%) all grades and grade 3 in 3 patients. Diarrhea (33%, grade 3/4 in 6%) and nausea (28%, grade 3/4 in 5%) were the most frequently observed gastrointestinal toxicities. Thromboembolic events occurred in 12 patients (15%) all grades and grade 3 in 8 patients (10%). No grade 4 thromboembolic event occurred. Overall, the combination of capecitabine and bevacizumab was generally well tolerated and the majority of adverse events were of mild to moderate intensity.

**Table 3:** Toxicity according to National Cancer Institute common toxicity criteria version 3

**Adverse event**	**All grades**		**Grade 3/4**	
**(safety population n = 78)**				
	**pts (n)**	**%**	**pts (n)**	**%**
Leucopenia	2	2	0	0
Anemia	4	5	1	1
Thrombocytopenia	4	5	1	1
Infection	29	37	6	7
Fatigue/Asthenia	20	25	1	1
Diarrhea	26	33	5	6
Mucositis	14	18	1	1
Nausea	22	28	4	5
Vomiting	9	12	1	1
Anorexia	8	10	1	1
Hand-foot-syndrome	44	57	16	21
Gastrointestinal perforation	2	2	2	2
Hemorrhage	10	13	1	1
Hypertension	17	22	3	4
Thromboembolic events	12	15	8	10

*Abbreviation*: pts (n) number of patients.

There were only 6 patients (8%) who experienced grade 4 adverse events, namely hematological toxicity, diarrhea, ileus, gastrointestinal perforation, blood infection and small bowel infection in one patient each. The 60-day mortality based on 78 evaluable patients was 3.8% (n = 3) and is within the expected range for this patient population.

## Discussion

Randomized clinical studies in patients with metastatic colorectal cancer have shown that bevacizumab improves response rates, progression-free survival and overall survival when combined with standard fluoropyrimidine based chemotherapy compared with chemotherapy alone [5,10,12,16,18,19]. Thus, bevacizumab in combination with chemotherapy (combination or single agent) has become a standard first-line treatment for patients with metastatic colorectal cancer.

Upfront stratification of patients according to patients’ and disease characteristics and the respective treatment aims seem to be of importance for the overall outcome and is reflected by current guidelines. Single agent or two drug regimens with fluoropyrimidines are recommended for patients presenting with non-resectable and/or asymptomatic disease, and/or co-morbidity, excluding from intensive first line chemotherapy or later surgery [9]. Besides clinical grouping according to the above-mentioned criteria, age and frailty are used for upfront patient stratification, although particularly frailty is not well defined. The FOCUS 2 trial included patients based on these criteria, who were randomized to fluoropyrimidines with or without oxaliplatin (with reduced starting dose), showing the feasibility and the beneficial impact of the combination regimen [20]. The recently reported phase III AVEX trial included patients of at least 70 years of age, deemed no optimal candidates for upfront irinotecan or oxaliplatin based chemotherapy, whereas the phase III AGITG-MAX trial included patients independent of age suitable for first line single agent [12,16]. Patients were randomized to capecitabine with or without bevacizumab (+/− mitomycin in AGITG-MAX). In both trials, the combination of capecitabine and bevacizumab resulted in significant and clinically meaningful improvement of PFS and showed a favourable ORR and OS compared to single agent capecitabine. Interestingly, all randomized trials with one of the somewhat less intensive chemotherapy backbones (i.e. IFL bolus regimen, 5FU/LV bolus regimens; capecitabine) showed consistently an impressive improvement of PFS (HR 0,54; 0,50 and 0,63 respectively) when bevacizumab was added to that backbone [10,12,19].

The here reported AIO KRK 0105 trial included patients, deemed to be unresectable independent of co-morbidity, age, symptoms or appropriateness for intensive first line chemotherapy. Median PFS seemed to be better in the AVEX and AGITG-MAX trials (9.1 and 8.5 months) compared to AIO KRK 0105 (7 months). Besides general limitation of a single arm phase II trial, patient selection and thus included patient population differed between the trials. Although overall patient characteristics (e.g. median age) were similar between the mentioned trials, some relevant differences were noted. The relatively high rate of symptomatic patients in the AIO KRK 0105 with 62% of patients with at least ECOG 1, compared to 48% or 44% in the AVEX and AGITG-MAX trials and the high rate of synchronous metastases in 72% of patients indicate a patient population with adverse prognostic features and high tumour load. Moreover, treatment duration, applied dose of capecitabine and subsequent treatment might have impacted on the different outcomes.

Median treatment duration of capecitabine and bevacizumab in the AIO KRK 0105 was 4.1 months, compared to 5.8 in AVEX and about 7 months in AGITG-MAX. The lower dosage of capecitabine (2 g/m^2^) in the AVEX trial and in about two thirds of the AGITG-MAX trial patients’ and thus a better and sustained tolerability might have been the reason for the longer treatment duration. However, besides the shorter treatment duration the higher dosage of capecitabine with 2.5 g/m ^2^ in the AIO KRK 0105 was well tolerated, particularly in regard of only 6% grade 3/4 diarrhoea.

Interestingly, second line chemotherapy was applied more often in the AIO KRK 0105 trial compared to the AVEX trial (57 vs. 37%). Moreover, rates of subsequent treatment with oxaliplatin (35 vs. 1.4%, AIO KRK 0105 vs. AVEX) or irinotecan (43 vs. 6%) highly differed. In the MAX trial only 17% in the capecitabine and bevacizumab arm received irinotecan and oxaliplatin in subsequent treatment lines.

Despite rarely used second line chemotherapy, the median PFS of 9.1 months resulted in a median OS of 20.7 months in the AVEX trial. It might thus be speculated, whether first-line treatment of bevacizumab in combination with capecitabine might preferably be used in elderly patients with rather indolent disease and a low chance of receiving subsequent treatment (assumed AVEX population) and maybe not ideally as initial treatment in patients with symptoms due to higher tumour load and/or worse prognostic features (e.g. synchronous disease), who are eligible for irinotecan and oxaliplatin-based chemotherapy (AIO KRK 0105 population).

However, first-line treatment of capecitabine and bevacizumab was well tolerated. Most adverse events were of mild to moderate intensity. The toxicity profile was as expected for the agents used. The most frequently observed adverse events were hand-foot syndrome, diarrhea, nausea, mucositis, fatigue, hypertension and thrombosis.

## Conclusion

Although the median PFS in the 78 patients who received study treatment was lower than expected and thus the primary study end point not met, the efficacy results of the trial are within the range of other capecitabine and bevacizumab combinations. Upfront patient selection and treatment stratification seem to be of utmost importance.

## Abbreviations

5FU: 5-fluorouracil; AE: Adverse event; AGITG: Australasian Gastrointestinal Trials Group; CEA: Carcinoembryonic antigen; CI: Confidence interval; CRC: Colorectal cancer; CT: Computed tomography; ECOG PS: Eastern cooperative oncology group performance status; EGFR: Epidermal growth factor receptor; EudraCT: European Clinical Trials Database; HR: Hazard ratio; KRAS: Kirsten rat sarcoma viral oncogene homolog; LV: Leucovorin; mCRC: Metastatic colorectal cancer; N: Number of patients; NCI-CTCAE: National Cancer Institute common terminology criteria for adverse events; ORR: Overall response rate; OS: Overall survival; P: P-value; PEI: Paul Ehrlich Institut; PFS: Progression free survival; PFSR@9: Progression free survival rate at 9 months; RECIST: Response evaluation criteria in solid tumours; SAE: Severe adverse event; ULN: Upper Limit of Normal; V: Version; Vs: Versus.

## Competing interests

The trial was funded by Roche. AS, DA, and SHB has received honoraria and research funding from Roche. The other authors declare that there is no conflict of interest.

## Authors’ contributions

AK and AS prepared the manuscript. DA was the coordinating investigators for the trial and participated in the preparation of manuscript and study protocol. DMB, TW, JZ, SH-B, EK, KP, and AK participated in patient recruitment. All authors read and approved the final manuscript.

## Pre-publication history

The pre-publication history for this paper can be accessed here:

http://www.biomedcentral.com/1471-2407/13/454/prepub

## References

[B1] JemalABrayFCenterMMFerlayJWardEFormanDGlobal cancer statisticsCA Cancer J Clin201161699010.3322/caac.2010721296855

[B2] FerlayJShinHRBrayFFormanDMathersCParkinDMEstimates of worldwide burden of cancer in 2008: GLOBOCAN 2008Int J Cancer2010127122893291710.1002/ijc.2551621351269

[B3] DouillardJYSienaSCassidyJTaberneroJBurkesRBarugelMHumbletYBodokyGCunninghamDJassemJRandomized, phase III trial of panitumumab with infusional fluorouracil, leucovorin, and oxaliplatin (FOLFOX4) versus FOLFOX4 alone as first-line treatment in patients with previously untreated metastatic colorectal cancer: the PRIME studyJ Clin Oncol2010284697470510.1200/JCO.2009.27.486020921465

[B4] Van CutsemEKohneCHLangIFolprechtGNowackiMPCascinuSShchepotinIMaurelJCunninghamDTejparSCetuximab plus irinotecan, fluorouracil, and leucovorin as first-line treatment for metastatic colorectal cancer: updated analysis of overall survival according to tumor KRAS and BRAF mutation statusJ Clin Oncol2011292011201910.1200/JCO.2010.33.509121502544

[B5] SaltzLBClarkeSDiaz-RubioEScheithauerWFigerAWongRKoskiSLichinitserMYangTSRiveraFBevacizumab in combination with oxaliplatin-based chemotherapy as first-line therapy in metastatic colorectal cancer: a randomized phase III studyJ Clin Oncol2008262013201910.1200/JCO.2007.14.993018421054

[B6] MaughanTSAdamsRASmithCGMeadeAMSeymourMTWilsonRHIdziaszczykSHarrisRFisherDKennySLAddition of cetuximab to oxaliplatin-based first-line combination chemotherapy for treatment of advanced colorectal cancer: results of the randomised phase 3 MRC COIN trialLancet20113772103211410.1016/S0140-6736(11)60613-221641636PMC3159415

[B7] BokemeyerCBondarenkoIHartmannJTde BraudFSchuchGZubelACelikISchlichtingMKoralewskiPEfficacy according to biomarker status of cetuximab plus FOLFOX-4 as first-line treatment for metastatic colorectal cancer: the OPUS studyAnn Oncol2011221535154610.1093/annonc/mdq63221228335

[B8] FalconeARicciSBrunettiIPfannerEAllegriniGBarbaraCCrinoLBenedettiGEvangelistaWFanchiniLPhase III trial of infusional fluorouracil, leucovorin, oxaliplatin, and irinotecan (FOLFOXIRI) compared with infusional fluorouracil, leucovorin, and irinotecan (FOLFIRI) as first-line treatment for metastatic colorectal cancer: the Gruppo Oncologico Nord OvestJ Clin Oncol2007251670167610.1200/JCO.2006.09.092817470860

[B9] SchmollHJVan CutsemESteinAValentiniVGlimeliusBHaustermansKNordlingerBvan de VeldeCJBalmanaJRegulaJESMO consensus guidelines for management of patients with colon and rectal cancer. A personalized approach to clinical decision makingAnn Oncol2012232479251610.1093/annonc/mds23623012255

[B10] KabbinavarFFSchulzJMcCleodMPatelTHammJTHechtJRMassRPerrouBNelsonBNovotnyWFAddition of bevacizumab to bolus fluorouracil and leucovorin in first-line metastatic colorectal cancer: results of a randomized phase II trialJ Clin Oncol2005233697370510.1200/JCO.2005.05.11215738537

[B11] KabbinavarFHurwitzHIFehrenbacherLMeropolNJNovotnyWFLiebermanGGriffingSBergslandEPhase II, randomized trial comparing bevacizumab plus fluorouracil (FU)/leucovorin (LV) with FU/LV alone in patients with metastatic colorectal cancerJ Clin Oncol200321606510.1200/JCO.2003.10.06612506171

[B12] TebbuttNCWilsonKGebskiVJCumminsMMZanninoDvan HazelGARobinsonBBroadAGanjuVAcklandSPCapecitabine, bevacizumab, and mitomycin in first-line treatment of metastatic colorectal cancer: results of the Australasian Gastrointestinal Trials Group Randomized Phase III MAX StudyJ Clin Oncol2010283191319810.1200/JCO.2009.27.772320516443

[B13] VrdoljakEOmrcenTBobanMHrabarAPhase II study of bevacizumab in combination with capecitabine as first-line treatment in elderly patients with metastatic colorectal cancerAnticancer Drugs20112219119710.1097/CAD.0b013e3283417f3e21057306

[B14] FeliuJSafontMJSaludALosaFGarcia-GironCBoschCEscuderoPLopezRMadronalCBolanosMCapecitabine and bevacizumab as first-line treatment in elderly patients with metastatic colorectal cancerBr J Cancer20101021468147310.1038/sj.bjc.660566320424611PMC2869164

[B15] PuthillathAMashtareTJrWildingGKhushalaniNSteinbrennerLRossMERomanoKWisniewskiMFakihMGA phase II study of first-line biweekly capecitabine and bevacizumab in elderly patients with metastatic colorectal cancerCrit Rev Oncol Hematol20097124224810.1016/j.critrevonc.2008.10.01219081732

[B16] CunninghamDLangIBevacizumab plus capecitabine versus capecitabine alone in elderly patients with previously untreated metastatic colorectal cancer (AVEX): an open-label, randomised phase 3 trialLancet Oncol201314111077108510.1016/S1470-2045(13)70154-224028813

[B17] TherassePArbuckSGEisenhauerEAWandersJKaplanRSRubinsteinLVerweijJVan GlabbekeMvan OosteromATChristianMCGwytherSGNew guidelines to evaluate the response to treatment in solid tumors. European Organization for Research and Treatment of Cancer, National Cancer Institute of the United States, National Cancer Institute of CanadaJ Natl Cancer Inst20009220521610.1093/jnci/92.3.20510655437

[B18] FuchsCSMarshallJBarruecoJRandomized, controlled trial of irinotecan plus infusional, bolus, or oral fluoropyrimidines in first-line treatment of metastatic colorectal cancer: updated results from the BICC-C studyJ Clin Oncol20082668969010.1200/JCO.2007.15.539018235136

[B19] HurwitzHFehrenbacherLNovotnyWCartwrightTHainsworthJHeimWBerlinJBaronAGriffingSHolmgrenEBevacizumab plus irinotecan, fluorouracil, and leucovorin for metastatic colorectal cancerN Engl J Med20043502335234210.1056/NEJMoa03269115175435

[B20] SeymourMTThompsonLCWasanHSMiddletonGBrewsterAEShepherdSFO’MahonyMSMaughanTSParmarMLangleyREChemotherapy options in elderly and frail patients with metastatic colorectal cancer (MRC FOCUS2): an open-label, randomised factorial trialLancet20113771749175910.1016/S0140-6736(11)60399-121570111PMC3109515

